# Creating a Culture to Avoid Knowledge Hiding Within an Organization: The Role of Management Support

**DOI:** 10.3389/fpsyg.2022.850989

**Published:** 2022-03-22

**Authors:** Sajjad M. Jasimuddin, Fateh Saci

**Affiliations:** ^1^Strategy, Entrepreneurship, and Sustainability Department, Kedge Business School, Marseille, France; ^2^Institut Paul Bocuse, Écully, France

**Keywords:** culture, knowledge hiding, knowledge hoarding, knowledge sharing, management support

## Abstract

Knowledge hiding is known to have negative consequences on organizational performance. The existing literature mainly focuses on the identification of antecedents and consequences of knowledge hiding. The studies pertaining to the top management role in creating a culture that stops concealing knowledge within an organization are limited. To fill that gap, the paper empirically address the knowledge sharing culture and to explore the management support to avoid knowledge hiding culture in an organization. This study based on an empirical study carried out in a United Kingdom-based laboratory within a high-tech global corporation, in which the atmosphere appeared conducive to knowledge sharing, and knowledge transfer appeared voluntary and spontaneous. The paper seeks to address why members of the case organization is reluctant about knowledge hiding among themselves. The study reveals that the management role is important in creating a culture that help discourage employees to withhold knowledge. The paper identifies the actions that top management takes to stop concealing knowledge within an organization. This study has provided several contributions. The findings of the study may be useful to managers and practitioners. For managers, this paper presents some important organizational factors that can be nurtured to avoid a knowledge-hiding culture in the organization. They can also take the management actions of the case organization as lessons to create a culture that encourage their employees to avoid knowledge hiding behavior.

## Introduction

Knowledge is widely considered to be a critical resource for an organization’s success, and the importance of knowledge transfer in supporting knowledge management initiatives is acknowledged (Jasimuddin, 2005; Jasimuddin et al., 2012; Zhang and Jasimuddin, 2015; Ruparel and Choubisa, 2020). Knowledge transfer is emphasized as a strategic issue for sustainable competitive advantage of an organization (Zhang and Jasimuddin, 2008; Jasimuddin and Zhang, 2009; Jasimuddin and Zhang, 2011). Contrarily, knowledge hiding is a counter-productive workplace behavior that has significant negative consequences on organizational performance (Huo et al., 2016; Jiang et al., 2019; Ellmer and Reichel, 2021; Xiong et al., 2021). Knowledge hiding was negatively associated with creativity of an organization (Černe et al., 2014; Rhee and Choi, 2017; Xiong et al., 2021). For example, in 2018, the losses associated with such behavior were reported to cost American organizations up to US$ 47 million in productivity (Nguyen et al., 2022). There is a tendency to hide knowledge, perhaps through fear of losing power or through uncertainty over job security (Jasimuddin et al., 2006). Resonate with this, Keong and Al-Hawamdeh (2002) observe that knowledge is power and no one is willing to give it away freely.

Knowledge hiding has been relatively a new topic of management research. The fact that prior knowledge management literature has focused mostly on knowledge sharing (Islam et al., 2018), and less on knowledge hiding (Arain et al., 2020a). Parallel to this, a limited literature is available in this domain (Xiao and Cooke, 2019; Arain et al., 2020b,^2021^; Ruparel and Choubisa, 2020). However, the studies pertaining to the top management role in creating a culture that helps discourage employees to hide knowledge are scant. Despite the general inclination of companies to have knowledge sharing culture, most employees attempt to conceal their knowledge (Ruparel and Choubisa, 2020). There is an ingrained policy prescribed by top management to encourage knowledge sharing practices. In general, employees refrain from practicing this in their workplace (Xiong et al., 2021). To the best of the authors’ knowledge, there is no research into the top management support in creating a culture to stop withholding knowledge within an organization. The study seeks to address the question of how top management actions help to create a culture that change knowledge hiding behavior of its employees.

Therefore, the paper attempts to explore the top management role in creating a culture that discourages knowledge hiding in an organization. The study offers several useful theoretical and managerial implications of the management support in discouraging knowledge hiding in organizations. The findings of the study may be useful particularly to managers and practitioners. For managers, this paper presents some important organizational factors that can be nurtured to create a knowledge-hiding-free culture in the organization. Interestingly, some novel constructs (e.g., patent rights, conference presentations etc.) have evolved from this study. These can encourage top management take into account to change knowledge hiding behavior of their employees.

The structure of the paper is as follows. First, the existing literature is reviewed so as to develop a theoretical basis for this research. Next, the methodology adopted in this study is outlined. The analysis of results are then presented, followed by the discussion of the empirical findings of the research. The paper concludes by reflecting on some of the implications of its findings for the theory and practice. Finally, the study limitations and future research direction are articulated.

## Literature

Knowledge sharing is a popular topic in knowledge management research (Jasimuddin, 2006; Jasimuddin et al., 2013). Knowledge hoarding and knowledge hiding are relatively new and under-researched topic (Connelly et al., 2012; Holten et al., 2016; Arain et al., 2020a). Recently, the phenomenon of knowledge hiding has increased the interest in researchers who have explored it in different views (Xiong et al., 2021). Several scholars treat it as deception (Takala and Urpilainen, 1999), knowledge withholding behaviors (Connelly et al., 2012) or counterproductive behaviors (Pearson et al., 2004; Xiong et al., 2021). Connelly et al. (2012) defined knowledge hiding as “an intentional attempt by an individual to withhold or conceal what has been requested by another person.” For the purpose of this study, knowledge hiding and knowledge hoarding are used synonymously.

A couple of review papers surrounding knowledge hiding is available. Ruparel and Choubisa (2020) systematically reviewed the relevant papers on knowledge hiding published between 2008 and 2018, arguing that these studies focus on the its antecedents as well as the consequences. Arain et al. (2020a) examines the consequences for innovative work behavior of top-down knowledge hiding – that is, supervisors’ knowledge hiding from supervisees. Similarly, Arain et al. (2021) identify the consequences of supervisor knowledge hiding in organizations based in Saudi Arabia. He et al. (2021) also provide another review of articles addressing the topic of knowledge hiding in organizations, showing that the central research themes of knowledge hiding include five clusters: concept and dimensions, antecedents, consequences, theories, and influence mechanisms.

Drawing on these reviewed articles, it is to be noted that the extant literature surrounding knowledge hiding is now enriched with the research that emphasizes on identifying its antecedents and exploring its negative consequences (Connelly et al., 2012, 2017; Černe et al., 2014; Fang, 2017; Butt, 2019; Butt et al., 2020). Parallel to this, (Butt et al., 2020) support this, stating that these studies mostly focuses on the antecedents and the consequences of knowledge hiding.

Most specifically, Xiong et al. (2021) did research into the antecedents of knowledge hiding and the social factors that trigger the relate behavior. Similarly, Butt et al. (2020) studied how knowledge hiding adversely affect buyer–supplier relationships, identifying the factors (i.e., limited interaction, mutual loyalty, and lack of interpersonal trust) that influence business relationship between managers of buying and supplying firms, when they conceal knowledge from each other.

Holten et al. (2016) investigated whether and how knowledge hoarding, functions as antecedent and consequence of work related negative acts, as a measure of bullying, with the use of mediation of trust and justice. Resonate with this, Arain et al. (2020b) examine the direct and indirect—*via* distrust in supervisor—relationships between supervisor knowledge hiding (SKH) and supervisee organizational citizenship behavior directed at the supervisor (OCB-S) in the context of the Middle East. They suggest that supervisees’ distrust in their supervisors mediates the significant and negative relationship between SKH and supervisees’ OCB-S. Parallel to this, Nguyen et al. (2022) show that role conflict, job insecurity, and cynicism positively impact knowledge hiding behavior, arguing that such behavior mediates the antecedents of knowledge hiding on job performance, and that transformational leadership moderated the impact of role conflict on knowledge hiding.

Issac and Baral (2018) argue that knowledge hiding is not meant to harm any other employee in the organization. But such action may lead to harm the company when it fails to get right knowledge at the right time in the right place to solve a problem or resolve a critical issue. The pervading culture of the case organization under study is not one in which employees feel the need to protect their jobs by hiding their knowledge. It is to be noted that the motivation of the knowledge contributor to provide knowledge is less straightforward (Jasimuddin, 2012). The top management definitely has a role to motivate employees to be so open and cooperative in sharing their knowledge with other organizational members. Hence, it is crucial to explore the top management support in creating a culture to stop withholding knowledge. As mentioned earlier, the study intends to fill this research gap by addressing the question of how top management actions help to create a culture that change knowledge hiding behavior of its employees. This paper investigates the management role underlying this phenomenon.

## Methodology

This research was carried out as an exploratory case study, which allowed to observe the phenomenon in a natural setting. Such an approach is widely used within the interpretive research paradigm, and is appropriate to explore social phenomena or contemporary events (Yin, 2004). The data collection and analysis procedure within in-depth qualitative research was based on the approach proposed by Miles and Huberman (1994). The research involved an in-depth case study of knowledge hiding practices in a United Kingdom-based laboratory within a high-tech global corporation.

The case organization, which is the one of the world’s biggest computer manufacturer, is responsible for numerous inventions, and regards knowledge sharing as an important part of its work. Respondents in the case organization report that organizational members are not worried about giving away knowledge to each other. Rather it appears that knowledge transfer is voluntary and spontaneous. In this study, data has been collected from interviews and observations. The interviews were tape-recorded and transcribed. The transcripts were coded to extract themes from the data. The themes were then interpreted to give a greater understanding of the case phenomena, as recommended by Miles and Huberman (1994). A sample of 30 interviewees was chosen purposively as Kuzel (1999) recommended that qualitative samples should be purposive rather than random. The employees based at the research laboratory requires to regularly collaborate with colleagues based in sites across the United States, France and the rest of the world to accomplish their assigned tasks. These interviews were more focused and theory-driven with what Miles and Huberman (1994) called “a well-bounded sample of persons”.

## Results

The empirical data has been analyzed to explore the top management actions to discourage knowledge hiding among employees within an organization. Knowledge hiding in the workplace is harmful. Organizations often make significant efforts to encourage employees to share knowledge (Xiong et al., 2021).

### Workplace – Collaborative, Open, and Discussion-Oriented

All the people interviewed in the organization under study recognize the value of knowledge transfer. The line managers encourage their colleagues to involve themselves in knowledge transfer processes so as to progress and get promotion. Technical mentors spend a lot of time transferring usual business matters to new entrants. Team leaders guide the employees working in their teams. The team leaders or technical mentors provide technical advice to their colleagues, particularly junior members, so that everybody could get up to speed and do their jobs properly. In this regard, a software developer remarks:

*“I am allowed to ask questions relating to my job. He [a team leader] volunteers to help me. He is one of my colleagues having more experience. We actually have technical mentor, team leader, immediate manager, and manager of managers [second line manager] to help us with technical advice.”*

Each member of a team has to pass on their knowledge to other peers within the functional group and to those who are working in other functional groups. An interviewee says, *“We are involved either in writing codes, testing them or whatever, I don’t think any of us can do so without sharing knowledge with others I guess.”* Parallel to this, a manager interviewed says, *“[the case organization], in my opinion, is an extreme example of corporate knowledge transfer [culture]. We are moving fast with the sharing of knowledge.”*

The employees interviewed at the research site are found to be quite collaborative and open. A software engineer notes: “*If he [to whom a question was asked] doesn’t know the answer then he turns around and tells me about others who might know. People are quite open to help each other out.”* The respondents report that they maintain very good relationships with their colleagues. For example, at lunchtime social meetings in the canteen, they discuss their job-related and customer-related issues. While having lunch with interviewees, the researcher notices that the interactions among the people appear cordial and job-focused.

Interviewees also appear cooperative as far as knowledge transfer is concerned. The respondents report that they never think that knowledge transfer would make them vulnerable and eventually translate into, for example, their job loss. A manager remarks: *“I don’t see anybody hiding back knowledge because we don’t think by transferring knowledge we will diminish in some way. I think it is natural thing; people are there just to do that [transfer knowledge]. There is no reason not to [transfer]. It is just part of what we need to do.”*

The Office layout of the case organization is kind of open plan. After several visits to the research site, the researcher finds a link between the seating arrangement and knowledge-sharing environment. At the case organization, two to three employees sit and work together in a single office room. There is rationale of keeping the open plan office. The majority of the people interviewed report that they prefer to work in an open plan environment, and some report that they feel bored working alone in a room. They like to interact during their work with others, particularly the members of their own team. One member states, *“Working in a room with others helps me ask them for help if I really have any query.”* Such an open plan is perceived as conducive to carrying out the transfer of knowledge. As a team leader says, *“Three of us working in a room so we can see each other and work together, that is our real benefit for the knowledge transfer to take place.”*

It is observed that most of the employees at the laboratory are working in small office rooms, but some are working in real open plan environments. A team leader explains: *“Open plan, that is right, I mean I actually prefer to work in open plan office. It is because I want to get all the people around me in a room. If I have a problem then there is always someone to ask, and someone else is around for interaction. I think it is very important for knowledge transfer. Sometimes you need to ask someone something. In open plan, there is always someone to discuss.”*

One feature observed during the visits is the fact that all the doors are invariably found to be open during office hours. Keeping doors open carries an important message; people actually welcome others to come inside the room to ask something. A team leader states, *“Door open means I like to be interrupted”.* It is noticeable feature of the case organization atmosphere. As a software developer says: *“I can just walk down the corridor and see from outside whether the individual [prospective knowledge contributor] I am looking for is available or not. If he is there, I can ask directly whether he can spare time to help me now.”*

Keeping door opened carries a message that entails the invitation to other colleagues to ask a technical query and also reflects team spirit and trust amongst themselves. A manager points out that: *“Certainly keeping door open implies ‘I am interruptible’. Look now, it is closed [during the interview] I don’t expect anybody to come in and ask unless it is real problem and urgent. But generally ‘yes’ the door is open and I think it is the case for everybody else. Keeping doors open means ‘come in and ask me something’. If other’s door is closed means ‘I don’t want to be disturbed’.”*

### Management Actions to Avoid Knowledge Hiding Within an Organization

There is a need to gain top management support to create a culture where employees spontaneously reluctant to withhold knowledge within the organization to do the job. Raub and Wittich (2004) supports this, arguing that “gaining support from line mangers” is crucial in this regard. Interviewees perceive management actions support to have a strong knowledge-sharing culture.

The management pays special attention to understand individuals’ attitudes toward knowledge transfer and knowledge hiding during the recruitment and selection process. Along with other qualities, e.g., education, skills and experience, of the applicants, their willingness to work in a team and their attitudes toward knowledge transfer are also considered at the time of hiring. A manager of managers (second-line manager) elaborates: *“It is because we hire those people who we find will transfer their knowledge. And the way in which the people are hired and trained helps to indoctrinate them not to hide and hoard knowledge.”*

From a managerial perspective, the respondents identify six aspects of management actions which help avoid knowledge hiding tendency of an employee.

#### Active Encouragement

The management basically encourages its members to carry out the transfer of knowledge for corporate benefit (e.g., Nielsen and Ciabuschi, 2003). Interviewees report that the management does not want to see one person emerging as the only expert in a particular field. Because there is no guarantee that the person will stay forever. If the person possessing the knowledge is not available for any reason, e.g., on holiday or sick, others will be stuck. So the management keeps discouraging its employees to conceal knowledge from other members by creating an environment. As a result, the people were found tol be reluctant in hiding their knowledge voluntarily. A software developer working in the WebShare Department remarks:

*“My manager periodically reminds us to make sure that our knowledge is available in written form*. *If someone is on holiday, his absence will not hamper others from carrying out his work. It should be there in the TeamRoom [interactive knowledge storage device within Lotus Notes]. Anyone within the TeamRoom can go to it, and do his [the person on holiday] job.”*

#### Incentives

Respondents have mixed views on incentives. One manager reveals, *“In my experience there is specific incentive.”* Contrarily, a team member reports, *“Management’s incentive*, *oh yes. But I can’t find any formal incentive* Another software engineer states, *“I think managers recognize people who help others. It is considered as a part of the culture and job, we try to share information [knowledge] as much as we can.”* However, there are indirect financial reward as incentives. A team leader points out: *“Certainly. [the case organization] likes those people who talk to their peers, talk publicly.* …*Unfortunately, I am not one of them. If an employee talks about what he is doing, then management recognizes that, there is financial reward not directly but in some way like promotion.”*

The managers keep assessing how interactive an employee is with other members of the team or organization, sometimes asking other members of the team how helpful a particular individual is. A team leader states, *“Management will ask the whole team about everybody else.”* There is a point system that is allocated for knowledge transfer as a part of performance appraisal. This supports the argument that the management is keen to see the employees do not hide knowledge.

#### Patent Rights

The case organization is very proud of its patent rights, which are thought to be the outcome of its members’ relentless efforts. So the software developers are encouraged to submit patentable ideas which are seriously taken into consideration for promotion to senior positions. While describing her experience, a manager mentions: “*If you give some idea which speeds up our work, I think you get recognition for this. Not for the usual business stuff. Clever ideas which people may start to use. We have a lot of recognition, particularly if you can bring brand new ideas, then apply for a patent or something like that. Informally, your manager will be pleased. There is lot of informal recognitions.”*

#### Supporting Conference Attendance

The employees are also encouraged to give talks at conferences, both inside the organization or outside. Attending conferences and presenting papers at top conferences such as Hawaii International Conference on System Sciences (HICSS) is highly appreciated by the management. As a team leader states, *“If I say ‘I would like to present a paper in a conference’, my manger will never say ‘no’.”* Rather the management provides logistic and financial support to make sure the person can attend the conference.

#### Publishing Papers

Furthermore, publishing paper(s) in scientific journals receives high recognition. A manager states, *“If you publish things, then [you] get some benefits [career progression].”* A couple of interviewees report that several colleagues have already produced papers, and published them in renowned journals. Although management support varies, the overall culture is for innovation and that is the message that comes from the higher level. A second-line manager explains: *“They [management] reward us for publishing [scientific papers]. It is seen as innovation. And there is a very keen culture for innovation. We want to be seen as innovative. We know that in order to keep moving forward we need to innovate. And publishing is counted amongst that.”*

There are scientific journals which demand Article Processing Charge (APC) for publishing articles. There is fund allocation from the company to pay the APC fee (directly to the publisher) by the management for accepted manuscript publication. Moreover, the management always encourages them to put things on the intranet so that others can benefit. The employees who post material also get recognition from the management, because they have written down something that can be used later on by others.

#### Career Progression

The majority of the interviewees report that managers promote those employees who do not hide knowledge; rather transfer knowledge to other colleagues. A team leader states, *“Potentially if you are looking for senior posts, it [promotion] is a very big motivation not to conceal knowledge.”* It is observed that rapid promotion is a tangible sort of incentive that an employee can expect. The more the engagement an individual has in knowledge share, the quicker the promotion he may expect. A manager tells a story about his promotion: *“I don’t think immediate financial help except you get promotion. If I look at [the case organization] and look at the people up there, they engage in sharing knowledge. I think it has been recognized. I think that is the way that helped me to get promotion. So it is not like that ‘you did this so this is your money for that.’ But my career progression happened because I was much more open [not withholding knowledge] than other people.”*

The interviewees perceive that the involvement in knowledge hiding is considered as a critical element in job evaluation of the people working at the case organization. A software engineer says, *“I think managers are aware of somebody who talks publicly and helps others with a technical advice.”* It becomes a part of the managers’ jobs to monitor their team members. One organizational member elaborates: *“Yeah. There is. Our management assesses people annually; we also have regular feedback sessions with people obviously. If an employee is seen interacting well and help others to share his knowledge then he is more likely to get recognition and eventually promotion. So it is not only helping the people in my team but also people across the boundaries*.”

## Discussion

Knowledge transfer is widely recognized as crucial for an organization’s survival (Argote et al., 2000; Jasimuddin et al., 2015; Islam et al., 2017). Whereas knowledge hiding is diminishes the creativity of an organization (Černe et al., 2014; Rhee and Choi, 2017). Organizations often make significant efforts to encourage employees to share knowledge. The fact that employees engage in knowledge hiding behavior to preserve their indispensability and career prospects (Butt et al., 2020). Parallel to this, Serenko and Bontis (2016) comment that knowledge hiders’ narrow-minded intentions urge them to intentionally hide knowledge from their colleagues. Whereas the most powerful employees in the future of an organization will be those who do the best job of transferring knowledge to others (Bilginoğlu, 2019). The management’s active support is essential to encourage organization members to engage in knowledge transfer activities and to create a culture that is conducive to knowledge transfer (Gupta and Govindaranjan, 2000; Nielsen and Ciabuschi, 2003; Islam et al., 2015). Nielsen and Ciabuschi, 2003), for example, contend that the management actively participates to encourage employees to engage in knowledge transfer. In this regard, Tang et al. (2015) argue that perceptions of employees about a leader being ethical keep employees from hiding knowledge.

Knowledge transfer culture is a precondition for successful knowledge management initiatives in organizations (Leidner, 1999; Jasimuddin and Zhang, 2014; Hasnain et al., 2016). The majority of the interviewees at the case organization report that they are engaged in transferring knowledge spontaneously. Almost all respondents mention that the company do have a strong knowledge-sharing culture. The organization under study has a culture where employees are directly discouraged to hide knowledge. The respondents consider knowledge transfer as being an important part of their job. The tasks and sub-tasks at the organization are interlinked in the sense that people cannot do their job properly without the help of other members of the organization. For example, a developer needs other developers’ technical help when he (she) engaging in writing software code. The interesting point is that the respondents view the corporate culture is very much knowledge sharing, collaborative and discussion-oriented.

The employees interviewed at the research site are found to be quite collaborative and open. Ipe (2003) reinforces this point of view by suggesting that “organizational values, such as openness, influence knowledge transfer activities”. Several other researchers (e.g., Hislop, 2005; Hasnain and Jasimuddin, 2012; Jasimuddin et al., 2014; Hasnain et al., 2016) also support this view by reporting that knowledge related values such as trust and openness have influence on knowledge transfer. The respondents report that they maintain very good relationships with their colleagues.

Discouraging its employees to participate in knowledge hiding is considered by the respondents as an important initiative of top management. New recruits are made aware of the negative impact of withholding knowledge from others. Several authors (Gupta and Govindaranjan, 2000; Jasimuddin, 2014) reinforce this point of view by suggesting that there is the relationship between knowledge sharing and incentives. Rather they are involved in knowledge transfer and, in turn, gives reward for doing so. This relationship between incentives and knowledge sharing is also further supported by Ipe (2003, p. 348) who argues that real and perceived reward and penalties for individuals come from sharing and hiding knowledge, respectively. Surprisingly, there is no direct penalty as an outcome for knowledge hiding at the case organization. However, management recognizes the value of knowledge sharing; one of the reported criteria for promotion at the organization under study is knowledge sharing.

Drawing on an empirical work in a large high-tech corporation, this paper identifies top management actions that helps avoid knowledge hiding. This supports the findings of Bilginoğlu (2019), who suggests that management should make the employees understand that there is more value in sharing knowledge than in hoarding it (Bilginoğlu, 2019). The study reveals that the top management role is important in creating a culture to stop withholding knowledge. This paper has taken a step toward the empirical identification of management actions, which might be seen as motivators to discourage knowledge hiding. The paper identifies management actions that helps avoid knowledge hiding behavior. Interestingly, some novel constructs (e.g., patent rights, conference presentations etc.) have evolved from this study. Top management gives recognition and promote to senior position if an employee can bring new idea, design and product, and then apply for a patent. The management provides logistic and financial support to make sure its employees can attend the conference and present a paper. These actions can encourage top management of other companies to take into account to change knowledge hiding behavior of their employees.

The paper is useful to managers and practitioners. Overall, this paper helps practitioners, particularly employers, in understanding the notion of knowledge hiding along with their role to discourage knowledge hiding behavior of employees. Most specifically, for managers, this study presents some important organizational factors that can be nurtured to create a knowledge-sharing culture in the organization. Having knowledge about the management support to discourage knowledge hiding may provide guidelines for working practices within an organization. It will help other companies to take these actions as a lesson. They can also take these lessons into practice to create culture that will change knowledge hiding behavior of their employees.

## Conclusion

Although the existing literature has stressed the causes and consequences of knowledge hiding, the management actions to discourage the knowledge hiding behavior of employees has not been fully or centrally addressed. This paper has filled this gap by exploring the top management support to create a culture to stop knowledge hiding tendency among employees, conducting research in a multinational corporation’s laboratory based in the United Kingdom. This paper reports that management has a role to create a culture that discourages knowledge hiding.

However, this study also has some limitations. Although the case organization is representative of a typical, mature high-tech multinational industry, the paper is based on insights from the existing literature along with the findings drawn from the single research setting. Hence, the results may not be generalized. As with other qualitative research approaches, the emphasis of this research is on the perceptions of the respondents. Although every effort is made to validate these, such a research approach is always open to multiple interpretations. To overcome this limitation, comparing the constructs of interest in other organizations from different industries would be a fruitful area for future studies. In addition, it might also be fruitful to consider comparative studies that may shed further light on the role of contextual features of organizations, such as size, culture and norms, which potentially can also influence on knowledge hiding. The fact that comparison with similar studies in other organizations will help to generalize in broader terms and explore similarities and differences between management actions against knowledge hiding practices. This paper lays some groundwork for future research particularly through further field studies in understanding the management actions in creating a culture that will discourage employees to hide knowledge within the organization.

## Data Availability Statement

The raw data supporting the conclusions of this article will be made available by the authors, without undue reservation.

## Author Contributions

Both authors listed have made a substantial, direct, and intellectual contribution to the work, and approved it for publication.

## Conflict of Interest

The authors declare that the research was conducted in the absence of any commercial or financial relationships that could be construed as a potential conflict of interest.

## Publisher’s Note

All claims expressed in this article are solely those of the authors and do not necessarily represent those of their affiliated organizations, or those of the publisher, the editors and the reviewers. Any product that may be evaluated in this article, or claim that may be made by its manufacturer, is not guaranteed or endorsed by the publisher.
